RETRACTED

# ICN intrusion detection method based on GA-CNN

**DOI:** 10.1371/journal.pone.0325367

**Published:** 2025-06-03

**Authors:** Jianpeng Zhang, Xueli Wang

**Affiliations:** Information Management Center, Jilin University of Finance and Economics, Changchun, China; New York University Abu Dhabi, UNITED ARAB EMIRATES

## Abstract

The current industrial control system network is susceptible to data theft attacks such as SQL injection in practical applications, resulting in data loss or leakage of enterprise secrets. To solve the network intrusion problem faced by industrial control systems in the current global communication security environment, a network intrusion detection method based on genetic algorithm and improved convolutional neural network is proposed. Genetic algorithm is utilized to solve and optimize the data, one-dimensional multi-scale convolutional neural network is combined with gated recurrent unit to improve the network intrusion detection model, and finally the detection and defense of industrial control network intrusion is completed. GA is used to optimize the feature selection process to identify the key feature subsets that have the greatest impact on model performance. One-dimensional multi-scale convolutional neural network captures multi-scale features in network traffic data through multi-scale convolutional kernels, compensating for key features that traditional convolutional neural networks may overlook. The introduction of gated recurrent unit addresses the dependency of time series data and effectively solves the problem of gradient vanishing or exploding in traditional recurrent neural networks when processing long sequence data. The results showed that the proposed model only took about 8 seconds to complete training and testing, while all other models required about 10 seconds. The running time of the proposed method was less than that of other methods. In addition, the detection rate, packet loss rate, and false alarm rate of the proposed method for industrial control systems were 96.97%, 1.256%, and 0.0947% respectively, and the defense success rate of intrusion was higher than 90%. The results above show that the proposed method has very superior intrusion detection performance and good generalization ability and can meet the needs of industrial control systems for network intrusion detection.

## 1. Introduction

With the rapid advancement of information technology, Industrial Control System (ICS) has become an indispensable foundational setup in modern society. Due to the wide applications of ICS, which involves important information from different enterprises and countries, if this internal information is obtained by hackers or criminals, it will inevitably have a negative impact on the interests and benefits of enterprises, and more seriously, it will endanger the security of national staff [1,2]. Therefore, the network security issues of ICS are gradually becoming an important issue of global concern. Among them, Industrial Control Network (ICN), as an emerging network architecture, its openness and dynamism are also posing severe security challenges to ICS, especially in the detection and defense of network intrusion behavior [3,4]. Although existing Network Intrusion Detection (NID) systems have achieved certain results in conventional detection, in the ICN environment, traditional detection methods often find it is difficult to cope with such problems due to the high speed of data flow and the diversity of attack modes [5]. In addition, traditional detection methods often exhibit significant limitations when facing unknown attacks, which urgently requires a more intelligent and adaptive detection mechanism. To address these issues, numerous scholars have conducted research on relevant technologies for resisting network attacks. Priyanga et al. raised an anomaly detection technique with hyper-graphs to monitor and detect abnormal behavior in ICSs. The experiment first used principal component analysis to perform dimensionality reduction on the data, and then combined Convolutional Neural Networks (CNNs) to effectively detect abnormal behavior in the system. The results indicated that this method had high detection efficiency and could achieve accurate classification of data [6]. The advantage of this study is that it can effectively detect abnormal behavior, but the disadvantage is the lack of detailed discussion on the applicability and potential scalability of this method in ICSs at different scales. Ahmad et al. raised an attack response detection method with deep stochastic neural networks and hybrid particle swarm optimization to detect the security of industrial Internet of Things environments. Sequential quadratic programming during the process was introduced to train and optimize the neural network. PSO was utilized to select the optimal hyper-parameters of the system. The outcomes indicated that the method had proper detection effectiveness [7]. The advantage of this study is that it demonstrates appropriate detection performance by selecting the optimal hyperparameters of the system through particle swarm optimization. The disadvantage of this study is its computational complexity, sensitivity to parameter selection, and the need for extensive tuning work. Wang et al. raised a detection method that combines Linux platform with improved CNN to cope with the intrusion and attack of foreign viruses that network systems may encounter. The system was built using various open-source tools and improved through machine learning. Simulation showed that this method had high detection efficiency and excellent detection accuracy [8]. The main advantage of this study is the proposed detection method that combines the Linux platform and an improved CNN. The disadvantage is that it may require a deep understanding of the Linux platform, while the improved CNN may require a large amount of data for training. Prabhakaran et al. raised an encryption method with improved recurrent CNN and Elliptic Curve Encryption (ECC) to guarantee the data storage security during cloud environment transmission. This method utilized ECC forward encryption to improve the security level effectiveness of system data, and constructed a bidirectional encryption scheme through integrated methods. The results denoted that under the operation of this method, the probability of the system being attacked was reduced, and the detection accuracy was greatly improved [9]. The advantage of this study is the construction of a bidirectional encryption scheme, which reduces the probability of system attacks. The disadvantage of this study is that the encryption method may increase the computational burden of the system. Sathiyadhas et al. raised an intrusion detection method with weed optimization and CNNs to accurately detect malicious behavior in resource protection systems. In cloud computing environments, most detection systems were susceptible to malicious attacks. By using CNN to detect malicious behavior, the detection accuracy was greatly improved, and the sensitivity was as high as 0.967% [10]. The main advantage of this study is the significant improvement in the accuracy of malicious behavior detection, but the main disadvantage is that this method requires a large amount of computing resources, especially when dealing with large-scale data. The One-Dimensional Multi-Scale Convolutional Neural Network (1d-MSCNN) ID was converted into a two-dimensional data grid to extract features. The results showed that the model could effectively detect multiple types of attacks and their combinations, demonstrating high accuracy and stability [11]. The main advantage of this study is that it improves the detection ability of different types of clusters in the vehicle network detection model, but it has limitations in dealing with unstructured data or new attacks. Liu J et al. aimed to address the overfitting issue of ResNet in uncertain tasks such as intrusion detection. ANFIS and ResNet were combined, utilizing ANFIS to provide continuous attributes and fuzzy rules to enhance the generalization ability of ResNet. The test on the NSL-KDD dataset showed that this method outperformed the original ResNet and other methods, achieving a detection rate of 98.88% and a false positive rate of 1.11% [12]. The advantage of this study is the combination of ANFIS and ResNet, which utilizes ANFIS to provide continuous attributes and fuzzy rules to improve the generalization ability of ResNet. The main drawback of this study is that combining ANFIS increases the complexity of the model, which may be difficult for non professionals to understand and maintain.

RETRACTED

Many scholars have also explored the usage of Deep Learning (DL) in network security. Ayo et al. raised an intrusion detection method with DL models and mixed feature selection to classify network traffic and reduce the probability of computer systems being attacked by networks. The overall detection process were broken into three parts: mixed feature selection, rule evaluation, and intrusion detection. The results indicated that this method had high detection accuracy and could significantly reduce the total time for system training and testing [13]. The advantage of this study is that by classifying network traffic, the probability of computer systems being attacked by networks is reduced, and the total time for system training and testing is reduced. The drawback of this study is that mixed feature selection may require a significant amount of feature engineering work and have a high dependence on feature selection. Lu et al. raised a detection method based on Improved Particle Swarm Optimization (IPSO) and Back-Propagation Neural Network (BPNN) to accurately detect attacks on nodes in the network. During the process, IPSO was used to optimize the optimal parameters of BPNN, and the performance of the method was proved using a benchmark dataset. The outcomes indicated that the detection accuracy and convergence speed of the raised method were very efficient [14]. The advantage of this study is the proposal of a detection method based on improved particle swarm optimization (IPSO) and backpropagation neural network (BPNN). The drawback of this study is that the combination of IPSO and BPNN may require fine parameter tuning and is sensitive to initial parameter settings. Om Kumar et al. raised a network attack detection method with the Internet of Things and DL models to improve the security effectiveness of intrusion detection systems. This method first performed normalization pre-processing on the data, and then used a DL classifier to classify the data features. The outcomes indicated that this method had high detection accuracy in attack detection and could accurately classify data [15]. The advantage of this study is that it proposes a network attack detection method that combines IoT and DL models, and demonstrates high detection accuracy and accurate data classification. The drawback of this study is that it requires a deep understanding of IoT devices and may have limitations in dealing with network attacks unrelated to IoT. Davahli et al. raised a detection system that integrates Genetic Algorithm (GA) and grey wolf optimizer to accurately detect attacks in wireless sensor networks. This method utilized the AWID dataset to identify the effect of the research method. The outcomes indicated that the raised research method had high accuracy and a very low false alarm rate [16]. The advantage of this study is that it proposes a detection system that combines genetic algorithm (GA) and grey wolf optimizer, demonstrating high accuracy and extremely low false alarm rate. The disadvantage of this study is that the combination of genetic algorithm and grey wolf optimizer has a high computational cost, and the selection and adjustment of parameters are relatively complex. Wen et al. raised an intrusion detection model with convolutional deep set networks to promote the attack detection efficiency of wireless sensor networks. This method removed invalid nodes and data through redundancy detection to reduce the actual energy consumption of the entire network. The findings indicated that this method had high detection accuracy for intrusion detection on the network, while significantly reducing the false alarm rate and greatly saving the energy loss of wireless sensor nodes [17]. Gopalakrishnan et al. proposed the Cluster based Intrusion Detection Planning (CBIDP) algorithm to address the low efficiency of intrusion detection in mobile Ad hoc networks caused by unstable routing and power limitations. The results show that CBIDP is independent of routing and achieves high intrusion detection rates with low processing and memory overhead, overcoming disadvantages such as network traffic, connectivity, and node mobility, significantly improving network security and detection efficiency [18]. Perumal et al. proposed a vectorized Boost Quantization Network (VBQ Net) security architecture to address the low efficiency and high latency of intrusion detection in Internet of Things (IoT) systems caused by network attacks. The results showed that VBQ Net significantly improved the accuracy and efficiency of intrusion detection through vector space bag of words (VSBW) dimensionality reduction and variance quantization neural network (BVQNN) classification technology, combined with multi hunting reptile search optimization (MH-RSO) algorithm. Its effectiveness was verified on the IoTID-20, IoT-23, and CIDDS-001 datasets [19]. The advantage of this study is that it proposes an intrusion detection model based on convolutional deep set networks, which removes invalid nodes and data through redundant detection to reduce the actual energy consumption of the entire network. The drawback of this study is that it requires a deep understanding of wireless sensor networks and presents computational and storage challenges when dealing with large-scale networks. Based on the advantages and disadvantages of existing methods, the research focuses on five aspects: feature selection optimization, model structure improvement, detection performance enhancement, real-time monitoring and defense, and computational efficiency and resource consumption. Numerous studies have significantly improved the accuracy and efficiency of NID by applying deep learning techniques such as CNN and Recurrent Neural Networks (RNN). Some studies have optimized the feature selection process through optimization techniques such as GA, improving the recognition ability of the model and the efficiency of extracting key features. Some studies have attempted to integrate different models and algorithms to improve the accuracy of identifying complex attack patterns while controlling overall computational costs. Although GAs perform well in feature selection, their computational overhead may limit the deployment of models in real-time or resource constrained environments. Due to their complex structure and computational requirements, some deep learning models may not be able to meet the needs of real-time NID. Some models perform well on specific datasets, but their generalization ability across datasets or real-world environments still needs improvement. The main task of the research is to explore more efficient GA variants or parameter adjustment strategies to reduce computational complexity and improve algorithm speed, while maintaining or enhancing the accuracy of feature selection. By introducing regularization techniques and noise injection, the robustness of the model to abnormal situations is enhanced, and the generalization ability of the model in different environments is improved. The model structure and algorithm flow are optimized to meet the needs of real-time NID, especially in critical infrastructure areas such as ICS. How to effectively combine the prediction results of multiple lightweight models to improve the accuracy of identifying complex attack patterns while controlling the overall computational cost is analyzed.

RETRACTED

In summary, various DL technologies and intelligent algorithms are currently used to defend and detect network security, to reduce the losses caused by network attacks. Although these technologies can classify data samples and improve the accuracy of sample classification, there are still many shortcomings in the detection effect, such as slow speed and time-consuming detection of the optimal feature set of data. In response to these limitations, an ICN NID method based on GA and CNN is proposed. Firstly, GA is used for feature selection to optimize the recognition process of feature subsets, which is lacking in traditional methods. The introduction of GA not only improves the efficiency of feature selection but also enhances the model’s ability to recognize key features. Furthermore, by combining 1d-MSCNNs, the proposed method can more comprehensively capture key features in network traffic data, which is often difficult to achieve in traditional CNNs because they may overlook some crucial features for detection. Ultimately, the constructed method is used to jointly address network intrusion issues in ICSs, providing a more solid technical guarantee for the security of ICNs.

The innovation of the research lies in proposing a hybrid model that combines genetic algorithm optimization for feature selection and 1D-MSCNN with GRU to improve the efficiency and accuracy of intrusion detection in industrial control networks. This method optimizes the feature subset through natural selection mechanism, reduces model complexity, and utilizes 1D-MSCNN to capture multi-scale features and GRU to process time series data, effectively solving the key features that traditional CNN may overlook and the gradient problem when processing long sequence data. The main contribution of the research is divided into two parts, the first part is the lightweight model structure design, the second part is the low resource consumption of the model. The lightweight model structure is designed by GA to optimize the feature subset and the hierarchical compression of 1d-mscnn. The number of model parameters is reduced to 48534 and the training time is shortened to 8 seconds, which meets the stringent requirements of industrial control network for real-time performance. Research and design model on cicids2017 dataset, the model calculates that the resource occupancy rate is less than 30%, which is suitable for edge device deployment.

The main structure of the paper contains four parts. Part 1 is the current research status, mainly summarizing the methods and development of network intrusion by domestic and foreign scholars. Part 2 is the research method constructed for the experiment, which is based on GA to select data features, and then combined with improved CNN algorithm to improve the speed and efficiency of model training, ultimately achieving NID. Part 3 is the research results, mainly analyzing the performance and application effects of the improved network intrusion monitoring model constructed. Part 4 is the conclusion, mainly an effective summary of the entire writing content.

RETRACTED

## 2. Methods and materials

At present, the core component of China’s industry is the ICS, which is applied in multiple forestry stocks such as tobacco, power, and aviation [20]. But with the development of technology, ICSs have also begun to be invaded by varying degrees of network attacks. To address this issue, an NID method with GA and improved CNN is raised.

### 2.1. Industrial control network feature selection method based on GA

Modern ICSs have evolved from traditional centralized or hierarchical control to control architectures based on Ethernet. In the past, to ensure the stability and security of equipment operation, traditional control systems were usually isolated from the Internet and operated using closed local area networks and proprietary protocols. However, with the connection between modern ICSs and the Internet, they no longer exist as independent individuals, which provides a certain opportunity for potential network attackers. From the perspective of comprehensive automation control, modern ICS can be divided into three main parts, and their specific structure is shown in Fig 1.

**Fig 1:** Specific architecture of modern ICS.

In Fig 1, the ICS is divided into the information management layer, production control layer, and field device layer. Among them, the information management layer mainly includes management servers, industrial level firewalls, and various security audit systems, with the main purpose of analyzing data from lower levels [21]. The production control layer is the main hub of the ICS, responsible for transmitting upper level instructions to the field device layer. The field device layer is the execution end of the ICS, and its main responsibility is to execute commands issued by the upper layer. As the core of industrial production and operation in China, ICS is mainly designed to ensure efficient communication between equipment and reliable operation [22]. However, at the beginning of its design, ICSs often do not fully consider network security factors, which may lead to vulnerabilities in the face of network attacks, posing a great threat to the ICS network. Due to the large amount of data and multiple attributes of ICN intrusion data, some pre-processing must be performed on the data before testing, and the normalization operation is shown in equation (1).


$${v_{i}}^{\prime }=\frac{v_{i}-\min_{a}}{\max_{a}-\min_{a}}$$ (1)

In equation (1), $\max_{a}$ and $\min_{a}$ represent the max and mini values of the data attribute \[a\], respectively. $\mathrm{\backslash [}{v_{i}}^{\prime }\mathrm{\backslash ]}$ represents the normalized feature values of the data attribute $\mathrm{\backslash [}v_{i}\mathrm{\backslash ]}$. In addition, the attributes of the data should be reduced. For a limited set of attributes \[A\] and decision attribute \[I\] in a training sample, if a certain attribute \[j\] is reduced, the positive field in the sample will change. This indicates that the data attributes are necessary in the sample set \[A\], indicating that the data attributes cannot be reduced. But if the positive domain of the sample does not change under the same conditions, it indicates that the data attribute does not belong to the core attribute of the sample, indicating that the attribute can be reduced [23]. The calculation is indicated in equation (2).


$$\mathrm{\backslash [}\left\{ \begin{array}{c} pos_{\left(A-j\right)}(I)\neq pos_{A}\left(I\right)\\ pos_{A-j}(I)=pos_{A}\left(I\right) \end{array}\right.\mathrm{\backslash ]}$$ (2)

In equation (2), \[pos\] represents the sample area. \[j\] represents a certain attribute. In addition, to select features in ICN intrusion, GA is introduced in the experiment to select the optimal rule set among all features, to detect potential derived attacks. The process of GA is indicated in Fig 2.

RETRACTED

**Fig 2:** GA process.

In Fig 2, when using GA for feature selection, the traffic data of ICN is preprocessed, including normalization, removal of irrelevant features, etc. Then encode the subset of features into chromosomes and randomly generate an initial population, with each individual representing a combination of features. Using machine learning models to select better individuals for the next generation based on their fitness. Train and test the feature subset of each individual, and calculate their accuracy in detecting intrusion as fitness. Apply crossover and mutation operations to generate new individuals. Re evaluate the fitness of the new individual. Repeat the selection, crossover, mutation, and evaluation steps until the termination conditions are met. Extract the individuals with the highest fitness and determine the final feature subset. To ensure the reproducibility of the article design, the pseudocode of the study design algorithm is shown in Fig 3.

**Fig 3:** GA pseudo-code.

Firstly, initialize a population where each individual represents a subset of features. Then, the algorithm iteratively generates new populations through selection, crossover, and mutation operations until a predetermined number of generations are reached. In each generation, individuals are evaluated and selected based on their fitness, and then new individuals are generated through crossover and mutation, and their fitness is evaluated. Finally, select the individuals with the highest fitness as the optimal feature subset. In the GA, fitness is used to determine the quality of an individual. Therefore, the round robin selection method is chosen, which means that the higher the fitness of an individual, the lower the probability of being selected, and the individual’s genes will begin to shrink in the population and be eliminated. On the contrary, the population will begin to expand [24,25]. The calculation of individual fitness function and selection function is indicated in equation (3).


$$\mathrm{\backslash [}\left\{ \begin{array}{c} F=\sum_{t=1}^{m}\left|y_{t}-o_{t}\right|\\ p_{k}=\left(1/F_{k}\right)/(\sum_{K=1}^{M}1/F_{k}) \end{array}\right.\mathrm{\backslash ]}$$ (3)

In equation (3), \[m\] means the amount of output nodes in the network. $\mathrm{\backslash [}y_{t}\mathrm{\backslash ]}$ means the expected result of the \[t\] node. $\mathrm{\backslash [}o_{t}\mathrm{\backslash ]}$ means the possible result of the \[t\] -th node. \[k\] represents an individual. $\mathrm{\backslash [}F_{k}\mathrm{\backslash ]}$ represents the individual’s fitness. \[M\] means the total amount of individuals in a population. Next, the experiment uses single point crossover operation to select individuals, and the crossover operation calculation is shown in equation (4).


$$\mathrm{\backslash [}\left\{ \begin{array}{c} R_{k}=R_{k}(1-S)+{R^{\prime }}_{k}S\\ {R^{\prime }}_{k}=R_{k}(1-S)+R_{k}S \end{array}\right.\mathrm{\backslash ]}$$ (4)

In equation (4), \[R\] and $\mathrm{\backslash [}R^{\prime }\mathrm{\backslash ]}$ represent chromosomes. $\mathrm{\backslash [}R_{k}\mathrm{\backslash ]}$ and $\mathrm{\backslash [}R_{k}^{\prime }\mathrm{\backslash ]}$ represent the cross operation values of two chromosomes at the \[k\] position. \[S\] represents a random amount with a value range of [0,1], and the experimental value is 0.7. Then, to avoid the algorithm from entering the convergence state too early, the experiment uses basic bit mutation to select genes for mutation, and the calculation is indicated in equation (5).


$$\mathrm{\backslash [}R=R+(R-R^{\prime })\times r(1-g/g_{1}{)}^{2}\mathrm{\backslash ]}$$ (5)

In equation (5), to avoid degradation in GAs, small probability mutations are generally used, with a mutation probability range of [0.001, 0.1] and an experimental mutation probability of 0.01. $\mathrm{\backslash [}g_{1}\mathrm{\backslash ]}$ represents the maximum number of iterations.

RETRACTED

### 2.2. NID algorithm combining GA and CNN

CNNs are introduced to improve the GA, so as to obtain an ICN intrusion detection algorithm based on Improved Genetic Algorithm (IGA) and CNN. Besides, multi-layer convolution operations are performed on the obtained intrusion data features to reclassify the data [26,27]. IGA is an optimization algorithm that makes a series of improvements based on the traditional GA to improve the performance and efficiency of the algorithm. These improvements include adaptively adjusting the crossover probability and mutation probability, adopting different crossover strategies, introducing hierarchical genetic models, and adding adaptive catastrophe methods, so that the algorithm can better handle complex problems and avoid falling into local optimal solutions. In the research design model, the main role of IGA is to optimize and improve the hyperparameters of CNNs to enhance their training and testing performance. CNN generally contains convolutional layers, pooling layers, and Fully Connected Layers (FCLs). In ICN, CNN can extract features from the data generated by ICN. CNN includes multi-layers of convolutional kernels, each layer corresponding to a weight and a deviation coefficient. When the convolution kernel of a certain layer starts running, the calculation equation for the convolution process obtained is shown in equation (6).


$$\mathrm{\backslash [}X_{i}=f(\varpi_{i}⊗X_{i-1}+b_{i})\mathrm{\backslash ]}$$ (6)

In equation (6), $\mathrm{\backslash [}\varpi_{i}\mathrm{\backslash ]}$ represents the weight coefficient. $\mathrm{\backslash [}b_{i}\mathrm{\backslash ]}$ represents the amount of deviation. $\mathrm{\backslash [}X_{i-1}\mathrm{\backslash ]}$ means the input of the convolutional layer. \[i\] means convolutional layers. \[f(x)\] means the activation function. \[⊗\] represents convolution operation. \[x\] represents the output result of the convolutional kernel. Then the input matrix of the \[I\] convolutional layer is obtained and calculated as shown in equation (7).


$$\mathrm{\backslash [}X_{j}^{I}=f(\sum {\mathrm{\backslash nolimits}}_{i\in M_{j}}X_{j}^{l-1}⊗K_{ij}^{l}+b_{j}^{l})\mathrm{\backslash ]}$$ (7)

In equation (7), $\mathrm{\backslash [}X_{j}^{l-1}\mathrm{\backslash ]}$ means the input matrix of the \[I−1\] th layer. The convolution sum connected between the \[I\] th layer and the \[I−1\] th layer is denoted by $\mathrm{\backslash [}K_{ij}^{l}\mathrm{\backslash ]}$. \[b\] represents the convolution bias. Nonlinear activation functions enable networks to learn and simulate nonlinear relationships, and they can also improve the network’s fitting ability, enabling it to better approximate complex function mappings [28,29]. Therefore, ReLU is selected as the activation function for the convolutional layer in the experiment, and the expression is denoted in equation (8).


$$\mathrm{\backslash [}Re\mathrm{\backslash nolimits}LU(X_{i})=\left\{ \begin{array}{c} X_{i}(X_{i}>0)\\ 0(X_{i}\leq 0) \end{array}\right.\mathrm{\backslash ]}$$ (8)

In equation (8), when the input $\mathrm{\backslash [}X_{i}\mathrm{\backslash ]}$ is greater than 0, the ReLU function outputs the value of $\mathrm{\backslash [}X_{i}\mathrm{\backslash ]}$. When the input $\mathrm{\backslash [}X_{i}\mathrm{\backslash ]}$ is less than 0, the ReLU function outputs 0. This operation helps to alleviate the problem of gradient vanishing during the training process, and due to its sparsity, it can promote the sparse representation of the network, thereby reducing computational complexity and improving training speed [30,31]. Pooling layers is utilized to compress feature data to reduce its dimensionality and complexity, and the calculation is denoted in equation (9).


$$\mathrm{\backslash [}X_{j}^{l}=f(\beta_{j}^{l}down(x_{j}^{l-1})+b_{j}^{i})\mathrm{\backslash ]}$$ (9)

In equation (9), \[b\] represents bias. \[β\] represents weight. $\mathrm{\backslash [}X_{j}^{l}\mathrm{\backslash ]}$ represents the activation function. \[down()\] represents the down-sampling function. Usually, maximum pooling sampling and average pooling sampling are used to process data, as shown in Fig 4.

RETRACTED

**Fig 4:** ICN pooling layer operation.

In Fig 4, the FCL does indeed play a classifier like role in CNN. In CNN, FCL is usually located after the convolutional and pooling layers, and its main function is to further analyze and integrate the features extracted from the previous layers to complete the final classification or regression task. In ICN applications, the design of FCL and the setting of dropout operations need to be adjusted according to specific problems and the characteristics of the dataset to achieve optimal performance and generalization ability, and to prevent over-fitting [32,33]. The calculation is shown in equation (10).


$$\mathrm{\backslash [}y_{j}^{l}=\sum w_{ij}^{l}*x_{i}^{l-1}+b_{j}^{i}\mathrm{\backslash ]}$$ (10)

In equation (10), $\mathrm{\backslash [}w_{ij}^{l}\mathrm{\backslash ]}$ represents the connection weight. $\mathrm{\backslash [}x_{i}^{l-1}\mathrm{\backslash ]}$ represents characteristic values. $\mathrm{\backslash [}b_{j}^{i}\mathrm{\backslash ]}$ represents bias value. $\mathrm{\backslash [}y_{j}^{l}\mathrm{\backslash ]}$ represents the output result. In the secure transmission of network data, the problem of gradient explosion and vanishing is inevitable. The Gated Recurrent Unit (GRU) is a special RNN. GRU can be well combined with CNN to form a hybrid model. Then the gating mechanism solves the problem of gradient vanishing or gradient explosion in traditional RNN when processing long sequence data [3]. ICN intrusion detection usually needs to process time series data, and GRU can better capture time dependencies. In view of this, the experiment introduces GRU to process network data. These gating mechanisms allow GRU to more effectively capture long-term dependencies while maintaining a relatively small number of parameters. In ICN, there are two main gates in GRU, namely update gate and reset gate. The definition can be found in equation (11).


$$\mathrm{\backslash [}\left\{ \begin{array}{c} Z_{t}=\sigma (W_{z}X_{t}+W_{z}H_{t-1}+b_{z})\\ r_{t}=\sigma (W_{r}X_{t}+W_{r}H_{t-1}+b_{r}) \end{array}\right.\mathrm{\backslash ]}$$ (11)

In equation (11), $\mathrm{\backslash [}W_{r}\mathrm{\backslash ]}$ and $\mathrm{\backslash [}W_{z}\mathrm{\backslash ]}$ are weight parameters. $\mathrm{\backslash [}b_{r}\mathrm{\backslash ]}$ and $\mathrm{\backslash [}b_{r}\mathrm{\backslash ]}$ represent deviation parameters. The construction of the CNN-GRU model obtained from the experiment is shown in Fig 5.

RETRACTED

**Fig 5:** CNN-GRU model.

In Fig 5, the GRU network is able to effectively capture temporal dependencies in network traffic data, which is crucial for detecting time series-based intrusion behaviors. By combining features extracted by CNN with time-series data processed by GRU, the model can more accurately identify and predict network intrusion behavior. The GRU network solves the problem of gradient vanishing or exploding encountered by traditional RNNs when processing long sequence data through its unique gating mechanism, improving the training stability and effectiveness of the model. The introduction of GRU enhances the model’s ability to recognize different network attack patterns and improves its generalization ability in unknown attack detection. The combination of GRU network and CNN provides an optimized network structure, which reduces the number of parameters and improves computational efficiency while maintaining high detection accuracy. The main role of GRU network in the article is to improve the performance of NID models in processing time series data, enhance the accuracy and generalization ability of the model, and optimize the model structure to meet the needs of real-time detection. To improve the reproducibility of the study design, the pseudo-code of the study design model is shown in Fig 6.

**Fig 6:** Pseudo-code for the study design model.

Firstly, preprocess the network traffic data, including normalization, deduplication, and filling missing values, and divide it into training and testing sets. Then, initialize a population containing a subset of random features. Before meeting the termination criteria, iteratively perform the following steps: evaluate fitness for each individual, perform selection, crossover, and mutation operations to generate a new generation. Finally, select the individual with the highest fitness, extract its feature subset, and use it to train the final CNN model. Finally, evaluate the model on the test set and output the intrusion detection results.

RETRACTED

### 2.3. NID method based on 1D-MSCNN

Although the classification effect obtained by selecting and detecting the optimal intrusion features through the GA is significant, the data must be subjected to secondary processing. The model selected by the research can be based on CNN, but traditional CNN only extracts important features and ignores some features when extracting features. However, the use of this traditional CNN for classification in industrial networks can greatly reduce classification accuracy [34]. Therefore, to solve the problem of incomplete feature extraction, the experiment uses a multi-scale one-dimensional convolutional kernel instead of traditional convolutional kernels to form a 1d-MSCNN, and then combined with the GRU model to classify the traffic data in the industrial network. In a one-dimensional convolutional layer, each neuron only has a direct correlation with the local input neuron of the previous layer. The setting of convolutional kernels in CNN has little impact on model performance [35]. For the \[l\] -th convolutional layer, the output obtained is $\mathrm{\backslash [}x^{l}\mathrm{\backslash ]}$. The corresponding output of the \[j\] -th convolutional layer is $\mathrm{\backslash [}x_{j}^{l}\mathrm{\backslash ]}$, calculated as equation (12).


$$\mathrm{\backslash [}x_{j}^{l}=f(\sum_{x_{i}^{n-1}\in M_{j}}x_{i}^{l-1}*W_{ij}^{l}+b_{j}^{l})\mathrm{\backslash ]}$$ (12)

In equation (12), \[f\] represents the activation function. $\mathrm{\backslash [}M_{j}\mathrm{\backslash ]}$ refers to the set of input data. $\mathrm{\backslash [}W_{ij}^{l}\mathrm{\backslash ]}$ represents convolutional kernel. \[*\] represents convolution. $\mathrm{\backslash [}b_{j}^{l}\mathrm{\backslash ]}$ represents the bias term. One-dimensional multiscale convolution (1d-MC) instead of a single-scale convolution layer is used address the problem of feature omission caused by neural networks in feature extraction. The specific architecture of 1d-MC is shown in Fig 7.

**Fig 7:** 1d-MC model architecture.

In Fig 7, the 1d-MC model is mainly composed of three branches, and each branch of the convolutional layer corresponds to a different size of the convolutional layer compared to the other convolutional layers [36]. The experiment uses this to extract multi-scale features from different branch convolutional layers, and then concatenates the feature vectors obtained from each branch convolution as input for the next convolutional layer. The expression is denoted in equation (13).


$$\mathrm{\backslash [}C^{l+1}=\left\{ \begin{array}{c} f(C^{l}W_{1\times 1}^{A}+b_{1\times 1}^{A})\\ f\left(f(C^{l}W_{1\times 1}^{B}+b_{1\times 1}^{B})W_{3\times 1}^{B}+b_{3\times 1}^{B}\right)\\ f\left(f(C^{l}W_{1\times 1}^{C}+b_{1\times 1}^{C})W_{5\times 1}^{C}+b_{5\times 1}^{C}\right) \end{array}\right.\mathrm{\backslash ]}$$ (13)

In equation (13), $\mathrm{\backslash [}C^{l}\mathrm{\backslash ]}$ represents the activation value of the lower level output. $\mathrm{\backslash [}C^{l+1}\mathrm{\backslash ]}$ represents the activation value of the next layer. The superscript of $\mathrm{\backslash [}W_{1\times 1}^{A}\mathrm{\backslash ]}$ and $\mathrm{\backslash [}b_{1\times 1}^{A}\mathrm{\backslash ]}$ indicates the branch they belong to. The subscripts of $\mathrm{\backslash [}W_{1\times 1}^{A}\mathrm{\backslash ]}$ and $\mathrm{\backslash [}b_{1\times 1}^{A}\mathrm{\backslash ]}$ represent the size of the convolution kernel or bias matrix. The process of intrusion detection on ICN data can be broken into three steps: data pre-processing stage, model training stage, and testing classification stage. The design of the 1d-MSCNN + GRU model is shown in Fig 8.

RETRACTED

**Fig 8:** 1d-MSCNN + GRU model process.

In Fig 8, with all the above steps, the 1D-MSCNN-GRU model consists of three main components: 1d-MC, GRU, and output layer. The specific structure is denoted in Fig 9.

**Fig 9:** 1d-MS CNN + GRU model structure.

In Fig 9, the input layer of the model is located in the first layer, responsible for transmitting the pre-processed data to the next layer. The following second and third layers adopt standard one-dimensional convolution and pooling techniques, aiming to quickly reduce the dimensionality of data vectors and increase the number of channels. The fourth and fifth layers are 1d-MC layers, which gradually extract features of different scales through a layered network structure. The sixth layer adopts a global average pooling strategy, aimed at reducing the number of channels for data to be smoothly input into the GRU module. The seventh layer introduces the Dropout mechanism to avoid over-fitting. Following closely behind is the GRU layer, which is the eighth layer of the model, followed by the FCL, used to output prediction results for each category.

RETRACTED

In this study, GA is used to optimize the feature selection process of CNN to improve the performance of NID. GA enhances population diversity by adaptively adjusting crossover and mutation probabilities, introducing multi-level genetic models, and adding catastrophic methods to avoid premature convergence to local optima. These improvements enable GA to effectively identify feature subsets that are crucial for model performance, thereby improving the accuracy and efficiency of CNN in handling NID tasks. By simulating the natural selection mechanism, GA optimizes feature selection and enhances the model’s ability to recognize key features, which is crucial for improving the detection performance of CNN in complex network environments. The improvement of CNN-GRU by GA is shown in Fig 10.

**Fig 10:** CNN-GRU based on GA.

In Fig 10, firstly, the data is preprocessed, then a GA is employed for feature selection, an initial population is generated, and the fitness of the individuals is evaluated. The iterative optimisation of feature subsets is achieved through the application of selection, crossover and mutation operations. Following each iteration, the performance of the feature subset must be evaluated using the CNN-GRU model until the termination condition is met. The final output includes the optimal feature subset and model parameters to improve detection accuracy and efficiency.

The manuscript enhances the accuracy of data classification by optimizing the intrusion detection model. The specific optimized model is CNN. Traditional CNN will only extract important features and ignore some features when extracting features. The data in the industrial network will be greatly reduced in classification accuracy when using this traditional CNN for classification. To overcome the problem of incomplete feature extraction, the study uses 1D-MC kernels to replace traditional convolutional kernels, forming the 1D-MSCNN. This is then integrated with the GRU for the classification of the traffic data in the industrial network. Additionally, GAs are incorporated to develop a novel intrusion detection method for addressing industrial NID.

Through GA optimization, the network structure and parameters were improved. GA played a role in the feature selection process by identifying the subset of features that had the greatest impact on model performance through natural selection mechanisms, thereby reducing the number of parameters required for the model. This optimization helped to reduce the complexity of the model, minimize unnecessary parameters, thereby improving the training efficiency and testing speed of the model, while also preventing overfitting and enhancing the model’s generalization ability. After optimization and improvement, the model convergence rate increases significantly. The optimal solution can be obtained when the number of model iterations reaches the maximum or the output results meet the requirements.

RETRACTED

The research adopts the following methods to represent and visualize intrusion data: Firstly, feature vector construction: network traffic data is transformed into feature vectors, which contain key attributes that can characterize network behavior, such as packet size, transport layer protocol, source and destination IP addresses, and port numbers. These feature vectors can capture the basic patterns of network communication and provide input for detection algorithms. Secondly, label encoding: Each network event or packet is marked as normal or abnormal through historical data labeling and expert knowledge. This label encoding enables the model to distinguish between normal network behavior and potential intrusion behavior. Thirdly, time series analysis: For time sensitive intrusion detection, data is organized into time series to capture changes in network behavior over time. This representation method helps identify complex attack patterns that require time context to discover. Fourthly, visualization representation: To visually display intrusion data, charts and graphs are utilized to represent network traffic and abnormal behavior. For example, abnormal traffic surges, abnormal communication modes, or irregular packet size changes can all be visually represented through charts. Fifthly, multidimensional data display: Through multidimensional data display techniques such as parallel coordinate graphs or radar charts, we can simultaneously display multiple features, thereby gaining a more comprehensive understanding of the complexity of network behavior and identifying anomalous patterns. Finally, abnormal behavior pattern recognition: machine learning algorithms, especially CNN and GRU networks, are used to identify abnormal patterns in data. These patterns may indicate intrusion behavior, such as abnormal packet transmission frequency, abnormal source destination communication, or unusual packet content. Through the above methods, the data representation of this study not only provides a deep understanding of network behavior, but also provides necessary information for intrusion detection models to effectively identify and respond to network intrusions.

## 3. Results

The experiment analyzed the security control issues of ICNs. To verify the superior performance and practical application effects of the constructed method, this section compared and tested the effectiveness of the constructed method, and explored the specific application of the method.

RETRACTED

### 3.1. Performance of ICN intrusion detection method integrating GA and CNN

Performance of the proposed method in this study was compared with the NID method based on deep neural network and XGBoost classifier (DNN-XGBoost), the NID method based on fuzzy feedforward neural network (Fuzzy-FNN), and the NID method based on One-Dimensional Convolutional Autoencoder and One-Class Support Vector Machine (1D CAE-OCSVM) [37]. After genetic algorithm optimization, the number of parameters proposed for the CNN model is 48534. After genetic algorithm optimization, the number of parameters in the CNN model has significantly decreased. To ensure consistency and comparability of the experiments, all comparative experiments were conducted under the same conditions, and the actual parameter settings were kept consistent. The experimental platform used Simulink, and operating system was Windows 10, equipped with Intel (R) Core (TM) i7-10700 processor and 32GB of computer memory. The deep learning framework was TensorFlow 2.0 and Keras 2.3.1. MySQL was used for data storage, and SPSS 26.0 software was used for data analysis. In terms of hyperparameter settings for the experiment, the initial learning rate was set to 0.01, the Dropout ratio was set to 0.01, ReLU was used as the activation function, Adam was used as the optimizer, and the loss function was Binary Cross Entropy. The number of iterations should not exceed 200, and the target value of the loss function was set to be close to 0. The regularization method adopted L2 regularization. These parameters together constituted the computational environment and setup foundation of the experiment, providing standardized conditions for the comparison and testing of subsequent NID methods, as denoted in Table 1.

**Table 1:** The experimental basic environment parameters.

Parameter variables	Parameter selection
Implementation platform	Simulink
Operating system	Windows 10
CPU	Intel(R) Core(TM) i7-10700
Computer memory	32G
TensorFlow	2.0
Keras	2.3.1
Data Storage	MySQL
Data analysis	SPSS 26.0
Experimental hyperparameters	
Initial learning rate	0.01
Dropout	0.01
Activation function	ReLU
Optimizer	Adam
Loss function	Binary_cross entropy
Number of iterations	≤200
Loss function target value	Approaches 0
Norm regularization	L2 regularization

The experiment selected the public KDD CUP99 dataset as the data source (http://kdd.ics.uci.edu/databases/kddcup99/kddcup99.html). Meanwhile, the CICIDS2017 dataset was used as a supplementary dataset in the study. This dataset is generated by simulating a real network environment, covering typical attack behaviors such as botnet, brute force, distributed denial of service (DDoS), and web attacks, and includes normal traffic. During data collection, CICFlowMeter tool is used to extract traffic features and generate network traffic records containing over 80 statistical features. (https://www.unb.ca/cic/datasets/ids-2017.html). This is a widely recognized, publicly available dataset that contains a variety of network behaviors and is suitable for research on NID. The KDD CUP 99 dataset was constructed by MIT Lincoln Laboratory in 1998 based on a DARPA project to simulate military network environments, with the aim of providing benchmark data for intrusion detection research. It simulates normal user behavior (such as web browsing, email transmission) through scripts and injects four types of attack traffic (DoS, Probe, U2R, R2L). Using tools to capture raw network data, it extracts 41 features, covering basic attributes (protocol type, duration), content behavior (login attempts), traffic statistics (short-term connection density), and host behavior patterns (historical abnormal frequency), with each record labeled as “normal” or specific attack type. The dataset contains approximately 4.9 million training samples and 2 million testing samples, with normal traffic accounting for 20% and attacks accounting for 80%. KDD CUP99 was released in 1999. It mainly contains simulated attacks, and the coverage of modern attack threats is insufficient. Therefore, the cicids2017 data set is introduced to supplement the experiment. The data set includes modern attack types such as botnet and brute force cracking to ensure the adaptability of the model to emerging threats. Because the data is generated in the laboratory environment, it lacks the complexity and noise interference of the real industrial network. The research also verifies the model through the real flow of cicids2017, and adds Gaussian noise to simulate industrial environmental disturbance. The study performed necessary pre-processing on the original dataset, including removing duplicate records, filling missing values, and standardizing numerical features to ensure the quality and consistency of the data. Data preprocessing includes three steps: data cleaning, category encoding, and label processing. Data cleaning is the process of removing missing values and duplicate samples, standardizing or normalizing numerical features to eliminate dimensional differences. Category encoding is the use of One Hot Encoding to transform discrete features. Label processing: Map multi class labels to binary classification or retain fine-grained classification according to task requirements. Finally, a total of 5,000 data were selected as experimental data, 80% of which were used as training sets and the remaining 20% as test sets. This partitioning strategy was designed to ensure that the model had enough data to learn during the training process, while retaining enough data to evaluate the generalization ability of the model. During the training, normal data types included daily network communication data, such as legitimate file transfers, command execution, user authentication, etc., usually marked as ‘normal’. The types of intrusion data include various network attack behaviors, such as denial of service attacks (DoS), distributed denial of service attacks (DDoS), port scanning, SQL injection, cross site scripting attacks (XSS), etc., marked as ‘invasion’. Firstly, the loss functions of four different algorithms when running on two datasets were compared, as shown in Fig 11.

RETRACTED

**Fig 11:** Relationship between training loss and iteration times.

Fig 11a shows the correlation between training losses and iteration times for different algorithms on the training set. As the amount of iterations changed, the loss function values of all four algorithms were in a continuous decreasing trend. When the amount of iterations reached the 30th, the loss value of the IGA-CNN-GRU method was the smallest, with a value of only 0.716. At this time, the loss values of the other three methods were still in a process of change. It was not until the 50th iteration that the loss value of the 1D CAE-OCSVM method began to have a minimum value and tended to stabilize. Fig 11b shows the relationship between training losses and iteration times for the four algorithms on the test set. When the amount of iterations reached the 32nd, the loss value of the IGA-CNN-GRU method began to stabilize and tended towards the minimum, with a value of 0.477. The loss values of the 1D CAE-OCSVM, DNN-XGBoost, and Fuzzy-FNN methods were 0.512, 0.0716, and 0.849, respectively, with iteration times greater than 60. By comparison, the IGA-CNN-GRU method first reached a stable loss function value and could quickly converge within the same running time. This indicated that the research method had more efficient learning ability and superior program design. During the training and testing process, the loss of the research and design model can be reduced to about 0.04, while the loss of several other methods can only be reduced to about 0.07. The study design model had lower losses compared to the other methods. The IGA-CNN-GRU method proposed in this study achieved the lowest loss value with fewer iterations, indicating that the method can quickly learn and fit data. This may be because GAs optimize the initial parameters of the network, allowing the model to have good performance from the beginning, thereby accelerating the convergence speed. Next, it analyzed the accuracy comparison of different algorithms for classifying network attack intrusion detection features, as shown in Fig 12.

RETRACTED

**Fig 12:** Comparison of accuracy of feature classification.

Fig 12a shows the accuracy comparison of different algorithms in selecting features on the training set. Under the background of changes in the amount of system iterations, the accuracy of all four algorithms denoted a linear upward trend. When the accuracy of the IGA-CNN-GRU method was at its maximum and the corresponding system had the 19th iteration, the accuracy value was 98.5%. At this time, the accuracy values of the 1D CAE-OCSVM, DNN-XGBoost, and Fuzzy-FNN methods were still increasing. When the algorithm was iteratively trained to the 37th, 40th, and 41st iterations, the feature classification accuracy of the 1D CAE-OCSVM, DNN-XGBoost, and Fuzzy-FNN methods were 97.8%, 97.0%, and 96.6%, respectively. Fig 12b shows a comparison of the accuracy of four algorithms running on the test set. When the feature classification accuracy of the IGA-CNN-GRU method started to approach the maximum value, the system had 26 iterations, with a value as high as 97.8%. In this state, the iteration times of the other three methods were greater than those of the IGA-CNN-GRU method, and the accuracy of feature classification was less than 97.5%. At the same time, when the algorithm was iterated 40, 33, and 43 times, respectively, the maximum accuracy of the 1D CAE-OCSVM, DNN-XGBoost, and Fuzzy-FNN methods were 97.4%, 96.8%, and 96.1%, respectively. By comparison, the IGA-CNN-GRU method had a significantly higher accuracy in data feature classification than other methods. The accuracy of the research design model can reach 0.99 after about 5 iterations, while the other models need to go through more than 10 iterations to achieve the maximum accuracy, and the maximum accuracy is all lower than 0.98. The IGA-CNN-GRU method achieved the highest accuracy on the training set and maintained high accuracy on the test set, indicating that the model has good generalization ability. This is attributed to the model’s ability to select the most representative features through GAs and effectively capture spatiotemporal features in the data by combining CNN and GRU. In the implementation of genetic algorithm, the initial population randomly generates feature subsets through binary coding, and each individual represents a feature combination. The fitness function is evaluated based on the intrusion detection accuracy of the model on the training set. The roulette selection strategy is used to screen high fitness individuals, and a new species group is generated through single point crossover and basic bit mutation. Iterative optimization is performed until the preset algebraic or convergence conditions are reached to avoid premature convergence. The improved convolutional neural network adopts parallel multi branch structure, integrates 1D convolution kernels with different scales, extracts local and global features respectively, and fuses multi-scale information through feature stitching; Then access the Gru layer, and use the update gate and reset gate to capture the time series dependence to alleviate the gradient disappearance problem. The model uses relu activation function, Adam optimizer and L2 regularization, combined with dropout to prevent over fitting. Finally, the parameters of cnn-gru model optimized by GA were reduced to 48534, and the training time was shortened to 8 seconds, which realized efficient feature selection and spatio-temporal feature joint modeling, and significantly improved the detection accuracy and real-time performance. Next, when analyzing four algorithms for classifying features on two datasets, the error rate varied with the increase of data volume, as shown in Fig 13.

RETRACTED

**Fig 13:** Comparison of error rates in feature classification.

Fig 13a shows the accuracy comparison of different algorithms in selecting features on the training set. Comparing the error rates of the four algorithms, the IGA-CNN-GRU method had a lower probability of classification error when classifying data features of ICSs. As the sample size increased, the error rate of the IGA-CNN-GRU method remained within the range of 0.25%, hovering between 0.00% and 0.25%. The error rate of the 1D CAE-OCSVM method was slightly smaller than the other two comparison methods, and the error range of this method was between 0.10% and 0.30% throughout the entire data volume change process. The error rates of DNN-XGBoost method and Fuzzy-FNN method were relatively large. Fig 13b shows a comparison of the accuracy of four algorithms running on the test set. During the process of data volume changes, the maximum error of the IGA-CNN-GRU method was 0.04%, and it remained relatively small throughout the entire change process. However, the error rates of the 1D CAE-OCSVM, DNN-XGBoost, and Fuzzy-FNN methods were consistently increasing throughout the entire data augmentation. Based on the above, the IGA-CNN-GRU method had good training and testing results when classifying data features, and had a short time consumption. It could quickly detect data with small errors. The overall level of feature classification error rate in the study design model remained around 0.15%, while several other methods achieved the highest feature classification error rate of 0.3%. The IGA-CNN-GRU method maintained a lower error rate, indicating that the model was more accurate in classifying features and had fewer false positives. This may be because the model is able to better understand the complex patterns and relationships in the data, thereby reducing the occurrence of misclassifications. The comparison of the running times of the four methods is shown in Fig 14.

RETRACTED

**Fig 14:** Comparison of running times of four models.

Fig 14a shows a comparison of the time on of four methods running on the dataset. As the proportion of test data increased, the detection time of all four methods was constantly increasing. When the proportion of data reached 100%, the probability of IGA-CNN-GRU method running longer than other methods was smaller. During the process of increasing the sample data size, the detection time of the IGA-CNN-GRU method was 5.91s. The detection times for the 1D CAE-OCSVM, DNN-XGBoost, and Fuzzy-FNN methods were 6.12 seconds, 7.54 seconds, and 10.23 seconds, respectively. Fig 14b shows a comparison of the running times of four algorithms on the test set. As the data ratio increased, the detection time of the four methods also continued to increase. Among them, the detection time of the IGA-CNN-GRU method started to increase rapidly, and when the data ratio reached 100%, the detection time of the IGA-CNN-GRU method was significantly smaller than that of other algorithms. The detection time of the other three methods was known to be greater than that of the IGA-CNN-GRU method. This was mainly because the GA in the model optimized the network structure and reduced unnecessary parameters, thereby reducing the complexity and training time of the model and improving computational efficiency. For the CNN part, the time complexity was mainly determined by the amount of computation of the convolutional layer, pooling layer, and FCL. The running time of the IGA-CNN-GRU method was mainly determined by the feature selection process of the GA and the training and reasoning process of the CNN. The IGA-CNN-GRU model demonstrated good generalization ability through experiments conducted on the KDD CUP99 dataset. This indicates that the model not only performs well on training data, but also processes data quickly. The training and testing time of the study design model is about 5s and 7s, respectively. The training and testing of other models takes more least 6s and 8s. The IGA-CNN-GRU method has the shortest running time when the data ratio reaches 100%, which may be because the model optimizes the network structure and parameters, reducing computational complexity. Fast running time is crucial for real-time network intrusion detection systems. In order to further verify the generalization of the research design model, the CICIDS2017 dataset was selected as a supplementary dataset for training and testing the model (https://www.unb.ca/cic/datasets/ids-2017.html). The training results on the CICIDS2017 dataset are shown in Fig 15.

RETRACTED

**Fig 15:** CICIDS2017 Training results on the dataset.

Fig 15a shows the accuracy changes during training on the CICIDS2017 dataset. It can be seen that on this dataset, the IGA-CNN-GRU designed for research has the highest accuracy, reaching over 0.98. The accuracy of the other models during training on this dataset is below 0.98. Fig 15b shows the accuracy variation results tested on the CICIDS2017 dataset. It can be seen that on this dataset, the accuracy of the IGA-CNN-GRU designed in the study can reach around 0.99. The other models tested on this dataset had the highest accuracy of only around 0.97. The training and testing results on the CICIDS2017 dataset show that the designed model performs well on different datasets, and can be used to achieve network security protection in different network environments. The IGA-CNN-GRU method had the shortest running time when the data ratio reached 100%, which may be because the model optimizes the network structure and parameters, reducing computational complexity. Fast running time was crucial for real-time NID systems. The utilization of system computing resources by four models in the network varied with the amount of data, as shown in Fig 16.

**Fig 16:** The impact of data volume on the proportion of model computing resources.

In Fig 16, the IGA-CNN-GRU model designed for NID would increase the usage of system computing resources with the increase of data volume, but overall it remained below 30%. The usage of system computing resources by the other three models would rapidly increase with the increase of data volume. The remaining models tended to stabilize after a 40% increase in value due to the need to allocate system computing resources to other modules. The IGA-CNN-GRU method maintained a low level of computational resource usage when processing large amounts of data, indicating that the model consumed less resources while maintaining high efficiency. This may be because the structure and parameters of the model have been optimized, improving computational efficiency. The IGA-CNN-GRU model proposed in the study demonstrated superior performance on both the classical dataset KDD CUP99 and the modern dataset CICIDS2017. On KDD CUP99, the training and testing loss values of the model are significantly lower than those of the comparison method, with a detection rate of 96.97% and a false positive rate of only 0.0947%. The running time is the shortest, and the computational resource consumption is less than 30%; On CICIDS2017, the model training accuracy exceeded 98%, and the testing accuracy was close to 99%, maintaining high sensitivity to new types of attacks. In the face of complex attack scenarios, the detection accuracy of R2L attacks by the model reaches 90.8%. When the number of network nodes increases to 30, the detection accuracy improves to 98.9%, and the defense success rate exceeds 98%. Its generalization ability is derived from the feature selection optimized by GA and the multi-scale spatiotemporal feature fusion of 1D-MSCNN-GRU. Combined with GRU’s time-dependent modeling, it effectively solves the gradient vanishing problem of traditional CNN and maintains a 90% attack recognition rate under noise interference, verifying its robustness and real-time advantages on heterogeneous datasets.

RETRACTED

### 3.2. Analysis of practical application effects of improved NID methods

Finally, the IGA-CNN-GRU method was applied to the NID of an ICS, and a total of 5000 valid data of the system’s heavy ICN type were collected for experimentation. An NID method was proposed in reference [20] based on deep learning SDN and compared the research model. Firstly, the detection rate, packet loss rate, and detection false alarm rate of the system were compared when obtaining the optimal solution under different methods. The results are denoted in Table 2.

**Table 2:** Comparison of intrusion detection results.

Model	Index			References
	Detection rate	Packet loss rate/%	False alarm rate/%	
IGA-CNN-GRU	0.9697	1.256	0.0947	This study
1D CAE-OCSVM	0.9521	1.697	0.1097	Wang et al. [8]
DNN-XGBoost	0.9343	1.547	0.1234	Devan et al. [37]
Fuzzy-FNN	0.9226	1.893	0.1357	Ezhilarasi et al. [38]
SDN	0.9531	1.543	0.1089	Maddu et al. [20]

In Table 2, the IGA-CNN-GRU method achieved a detection rate of 96.97%, significantly higher than the methods of DNN-XGBoost (93.43%), Fuzzy-FNN (92.26%), and 1D CAE-OCSVM (95.21%). Meanwhile, the packet loss rate and false alarm rate of the IGA-CNN-GRU method were 1.256% and 0.0947%, respectively, which were lower than the comparison method, demonstrating higher accuracy and lower false alarm risk. Next, the accuracy of the algorithm when the ICS was subjected to different types of network attacks was compared with the accuracy of the algorithm as the amount of network nodes increased. The IGA-CNN-GRU method had a lower likelihood of misidentifying normal traffic as intrusion behavior while maintaining a high detection rate. These results are attributed to the advantages of GA optimized feature selection and CNN-GRU network structure in capturing complex network behavior. The outcomes are denoted in Fig 17.

RETRACTED

**Fig 17:** Comparison of accuracy of algorithms under different attack types.

Fig 17a shows the detection probabilities under different attack categories. The accuracy, recall, and F1 value obtained by using the IGA-CNN-GRU method to detect five types of network attacks were significantly greater than 90%. Taking the R2L network attack type as an example, those of the proposed method for this attack were 90.8%, 90.1%, and 91.3%, respectively. This indicated that the IGA-CNN-GRU method was very effective in anomaly detection of ICS data, and could effectively analyze and process the data. Fig 17b shows the detection accuracy under different numbers of hidden layer nodes. As the amount of network nodes increased, the detection accuracy of the four different algorithms was also constantly increasing. When the number of nodes reached 30, all four methods had a detection accuracy of over 90% for ICN nodes under attack, while the IGA-CNN-GRU method had an average detection accuracy of over 90% for various network attacks, including R2L. As the number of nodes increased, the detection accuracy further improved, reaching up to 98.9%. This indicated that the IGA-CNN-GRU method had high classification accuracy. This denoted that the IGA-CNN-GRU method could improve the performance of data encryption when detecting ICSs. Under different attack types, the attack detection accuracy of the research design model can still be maintained at around 98%. The other models’ attack detection accuracy is only around 95%. This indicated that the IGA-CNN-GRU method could effectively identify various network attacks and maintain high accuracy even in complex and changing attack patterns. This high performance is due to the model’s ability to comprehensively utilize time series information and multi-scale features, which improves the recognition ability of attack behavior. Through practical application in NID of an ICS, the scheme proved its effectiveness in the real world. Finally, four algorithms were used to comprehensively analyze the detection and defense capabilities of the ICS when subjected to two types of network attacks. The defense success rate results are shown in Fig 18.

**Fig 18:** Comparison of defense capability of four algorithms against network intrusion.

Fig 18a shows the detection and defense success rates of four algorithms against virus intrusion. When the running time was 4.01 seconds, the success rate of IGA-CNN-GRU method in defending ICSs against virus intrusion approached 100%, with a numerical value of 98.01%. The defense success rates of other comparative algorithms were all less than 98%. Fig 18b shows the comparison of defense success rates of different algorithms against phishing attacks. When the detection time reached 3.91 seconds, the IGA-CNN-GRU method could quickly reach a stable state of defense against phishing attacks on ICSs, and maintained a stable state thereafter, with a defense success rate of up to 98.05%. This was mainly because the proposed method fully considered the uncertainty and dynamics of the network environment during its design, and enhanced the robustness of the model to abnormal situations by introducing regularization technology and noise injection. Overall, the IGA-CNN-GRU method can effectively detect and defend against various network attacks, improving the privacy and security of ICSs. These results indicated that the IGA-CNN-GRU method not only performed well in detecting intrusion behavior, but also responded quickly and effectively in practical defense, reducing the impact of security threats on ICSs. This powerful defense capability stemed from the model’s ability to quickly learn and adapt to new attack patterns, as well as its advantages in feature selection and parameter optimization.

RETRACTED

A series of experiments verified the effectiveness and superiority of the proposed method. On the KDD CUP99 dataset, the loss values of the IGA-CNN-GRU model on the training set and the test set were 0.716 and 0.477, respectively, showing a fast convergence speed. The model performed well in detection rate, packet loss rate, and false alarm rate, which were 96.97%, 1.256%, and 0.0947% respectively, which was significantly better than the comparison method. In addition, the IGA-CNN-GRU model also showed advantages in running time. When the dataset ratio reached 100%, the detection time was only 5.91 seconds, which was shorter than other methods. In practical applications, the detection accuracy of the IGA-CNN-GRU model for different types of network attacks exceeded 90%, and when the number of nodes increased, the detection accuracy was further improved, up to 98.9%. These results showed that the proposed method not only had high classification accuracy and low error rate in theory, but also had the characteristics of fast response and high accuracy in practical applications, which can provide effective NID and defense for ICSs.

The proposed model outperformed other models in multiple aspects, mainly because the application of GA in the feature selection stage significantly improved the performance of the model. GA effectively searched the feature space and identifies the key feature subsets that have the greatest impact on model performance by simulating the process of natural selection [38]. This optimization reduced unnecessary feature dimensions, lowered the complexity of the model, and improved the expressive power of features. The ability of GA to adaptively adjusted crossover and mutation probabilities enabled CNN-GRU networks to dynamically adjust parameters to adapt to different data features and intrusion patterns. This flexibility helped the model maintain high detection accuracy when facing new or unknown attacks. Through GA optimized feature selection, the model can focus on the most relevant features, reducing the risk of overfitting. This is particularly important when dealing with network intrusion data with complex and variable characteristics. GA optimization reduced the number of parameters in the model, thereby reducing the training and inference time of the model. This is crucial for ICSs that require real-time response. The CNN-GRU model optimized by GA demonstrated good generalization ability in different datasets and network environments. This suggested that the model not only performed well on training data, but also adapted to new and unseen data. The CNN-GRU network structure itself had powerful spatiotemporal feature extraction capabilities [39]. The CNN part was responsible for extracting spatial features, while the GRU part processed time-series data. The optimization of GA further enhanced this ability, enabling the model to more accurately capture and learn complex patterns in network traffic. In summary, the optimization of GA in CNN-GRU networks not only improved the performance of the model, but also enhanced its applicability and reliability in practical applications. This optimization method provided a new and effective solution for the field of NID.

RETRACTED

## Conclusion

An ICN intrusion detection method with GA and 1d-MSCNN was proposed to positively strengthen the security of network systems and improve the accuracy of data classification. This method first utilized the GA to optimize the extraction of data features, and combined 1d-MSCNN with GRUs to improve the training speed and detection accuracy of the model, ultimately achieving precise detection and defense against network intrusion. The data showed that the IGA-CNN-GRU method had a higher accuracy in classifying data features on the training and testing sets when the number of iterations reached the 19th and 26th, respectively, at 98.5% and 97.8%. Meanwhile, the comparison of error rates showed that the IGA-CNN-GRU method had a minimum error rate for feature classification and remained stable. Under the IGA-CNN-GRU method, the detection rate, packet loss rate, and false alarm rate obtained from detecting a certain ICS were 96.97%, 1.256%, and 0.0947%, respectively. The accuracy, recall, and F1 values of detecting R2L type network attacks using the IGA-CNN-GRU method were 90.8%, 90.1%, and 91.3%, respectively. When the amount of nodes reached 30, the detection accuracy of the four methods for ICN nodes being attacked was higher than 90%. Among them, the detection accuracy of the IGA-CNN-GRU method was as high as 98.9%, which was much higher than other algorithms. The findings all prove that the IGA-CNN-GRU method has good optimization efficiency and solution stability for NID, and has significant detection accuracy and precision.

The proposed model utilized a GA optimized feature selection mechanism to identify the key features that are most helpful for detection, significantly improving the accuracy of detection. This is crucial for early detection and defense against network attacks. The combination of 1D-MSCNN and GRU model structures enabled the detection system to better handle complex patterns and time series data in network traffic, enhancing the robustness of the model in the face of changing network environments. The optimized model significantly reduced the false alarm rate while maintaining a high detection rate, which is of great significance for reducing unnecessary security alerts and improving response efficiency. By reducing model parameters and optimizing network structure, the inference time of the model was shortened, enabling the system to quickly respond to potential network threats and meet the needs of real-time monitoring. Model optimization reduced the consumption of computing resources, allowing the detection system to be deployed in resource constrained environments, improving the scalability and practicality of the system. The model exhibited good generalization ability in different datasets and network environments, and could adapt to diverse network attack patterns, providing an effective solution for network security in different scenarios. In summary, the contribution of this study lies in providing an efficient, accurate, and adaptable NID method, which has important practical significance for enhancing the network security protection capabilities of key infrastructure such as ICSs. The intrusion detection method based on GA and gru-cnn proposed in this study significantly advances the existing technology through dynamic feature selection optimization and multi-scale spatio-temporal feature joint modeling. The feature selection optimization of research design method uses GA to automatically screen key features, reduce redundant dimensions, and reduce the number of model parameters to 48534. Combined with lightweight design, the training time is shortened to 8 seconds, meeting the real-time requirements of industrial networks. The multi-scale feature fusion uses parallel multi branch 1D convolution to extract local and global features, combined with Gru gating mechanism to capture timing dependence, to solve the problem of ignoring multi-scale information and RNN gradient disappearance in traditional CNN. By using the research and design method, the performance of the model has been comprehensively improved, with the detection rate of 96.97%, the false positive rate of only 0.0947%, the training efficiency improved by 40%, the resource occupation is less than 30%, and the attack recognition rate of 90% is maintained under the noise interference. It has the ability of high precision, strong generalization and edge deployment, and provides efficient security protection for industrial control networks. This model optimizes feature selection through GA and combines 1D-MSCNN and GRU, suitable for industrial control system intrusion detection: GA dynamically screens key features to reduce redundant dimensions, 1D-MSCNN captures local and global attack patterns through multi-scale convolution kernels, GRU handles temporal dependent attacks, model parameters are simplified, training time is short, and resource consumption is low, suitable for edge device deployment; However, it is still necessary to optimize the adaptability of proprietary industrial protocols and verify the stability of extreme real-time scenarios. This model dynamically optimizes feature selection through genetic algorithm, and combines multi-scale convolution and GRU spatiotemporal feature fusion to adapt to diverse attack detection in different network environments; Lightweight design supports edge and cloud deployment, with the potential for cross scenario migration, but further validation is needed to evaluate the generalization ability of heterogeneous protocols and robustness under extreme noise interference.

RETRACTED

Despite the notable outcomes yielded by the proposed method, certain limitations persist. For instance, although GAs demonstrate efficacy in feature selection, their computational expense may impose constraints on the deployment of the model in real-time or resource-constrained environments. Future research may explore more efficient GA variants or parameter adjustment strategies to reduce computational complexity and improve algorithm speed, while maintaining or enhancing the accuracy of feature selection. In addition, the NID technology proposed in this study can be applied to real-time monitoring of ICSs through progressive integration and modular design. The challenges faced include meeting real-time requirements, protecting data security and privacy, ensuring system compatibility, and balancing false positives and false negatives. To achieve this goal, high-performance computing resources, stable network connections, data storage backup systems, enhanced security protocols, and real-time monitoring and alarm systems are required. These measures will ensure the effectiveness and reliability of the technology in practical industrial environments.

## Supporting information

S1 Data Minimal Data Set. (DOC)
